# Effect of lithium on ventricular remodelling in infarcted rats via the Akt/mTOR signalling pathways

**DOI:** 10.1042/BSR20160257

**Published:** 2017-03-27

**Authors:** Tsung-Ming Lee, Shinn-Zong Lin, Nen-Chung Chang

**Affiliations:** 1 Department of Medicine, Cardiology Section, An Nan Hospital, China Medical University, Tainan, Taiwan; 2 Department of Medicine, China Medical University, Taichung, Taiwan; 3 Cardiovascular Research Laboratory, China Medical University Hospital, Taichung, Taiwan.; 4 Division of Cardiology, Department of Internal Medicine, School of Medicine, College of Medicine, Taipei Medical University, Taipei, Taiwan; 5 Bioinnovation Center, Tzu Chi foundation; Department of Neurosurgery, Buddhist Tzu Chi General hospital, Tzu Chi University, Hualien, Taiwan; 6 Division of Cardiology, Department of Internal Medicine, Taipei Medical University Hospital, Taipei, Taiwan

**Keywords:** Echocardiography, Nuclear factor of activated T-cells, Physiological hypertrophy, Myocardial infarction, Ventricular remodeling

## Abstract

Activation of phosphoinositide 3-kinase (PI3K)/Akt signalling is the molecular pathway driving physiological hypertrophy. As lithium, a PI3K agonist, is highly toxic at regular doses, we assessed the effect of lithium at a lower dose on ventricular hypertrophy after myocardial infarction (MI). Male Wistar rats after induction of MI were randomized to either vehicle or lithium (1 mmol/kg per day) for 4 weeks. The dose of lithium led to a mean serum level of 0.39 mM, substantially lower than the therapeutic concentrations (0.8–1.2 mM). Infarction in the vehicle was characterized by pathological hypertrophy in the remote zone; histologically, by increased cardiomyocyte sizes, interstitial fibrosis and left ventricular dilatation; functionally, by impaired cardiac contractility; and molecularly, by an increase of p-extracellular-signal-regulated kinase (ERK) levels, nuclear factor of activated T cells (NFAT) activity, *GATA4* expression and foetal gene expressions. Lithium administration mitigated pathological remodelling. Furthermore, lithium caused increased phosphorylation of eukaryotic initiation factor 4E binding protein 1 (p-4E-BP1), the downstream target of mammalian target of rapamycin (mTOR). Blockade of the Akt and mTOR signalling pathway with deguelin and rapamycin resulted in markedly diminished levels of p-4E-BP1, but not ERK. The present study demonstrated that chronic lithium treatment at low doses mitigates pathological hypertrophy through an Akt/mTOR dependent pathway.

## Introduction

Ventricular remodelling is associated with cardiac physiological or pathological hypertrophy after myocardial infarction (MI), depending on interventional drugs [1]. Distinct signalling pathways are responsible for the development of cardiac pathological and physiological hypertrophy. Physiological hypertrophy is mediated primarily by the insulin-like growth factor-1/phosphoinositide 3-kinase (PI3K (p110α)) pathway [2]. Akt, a downstream target of PI3K, phosphorylates and activates the mammalian target of rapamycin (mTOR), which is central to cardiac physiological hypertrophy. Transgenics with a dominant-negative mutant of the PI3K subunit p110α or a disruption of the *Akt1* gene have virtually no signs of hypertrophy in response to exercise training [3], a kind of cardiac physiological hypertrophy. In contrast, pathological hypertrophy is mediated by G-protein-coupled receptors (GPCRs) following stimulation by hormones such as angiotensin II and endothelin-1, both of which are increased after MI [4]. Activation of GPCRs results in a number of downstream signalling events, such as activation of mitogen-activated protein kinases (MAPKs) (e.g. extracellular-signal-regulated kinase (ERK) 1/2 (ERK1/2)) and dephosphorylation of nuclear factor of activated T cells (NFAT) transcription factors by calcineurin [5]. NFAT is not activated by physiologic stimuli, suggesting that activation of NFAT may specifically regulate pathological remodelling of the myocardium [6]. Thus, the PI3K/Akt axis seems more linked to physiological hypertrophy, whereas MAPK signalling and NFAT pathways participate in the development of the pathological hypertrophy. Physiological hypertrophy shows a normal cardiac structure with a relatively normal pattern of cardiac gene expression and improved cardiac function [7]. Pathological hypertrophy is associated with cardiomyocyte hypertrophy, interstitial fibrosis, cardiac dysfunction, left ventricular dilatation and increased expression of foetal genes such as atrial natriuretic peptide (ANP), β-myosin heavy chain (β-MHC) and skeletal α-actin [8,9].

Lithium has been the mainstay of treatment for bipolar disorder for more than 60 years. Lithium has been recognized for its neuroprotective effects against diverse insults, such as ischaemia, both *in vitro* and *in vivo* [10,11]. Recently, lithium has been shown to activate insulin-like growth factor-1 [5], which in turn triggered PI3K/Akt signalling pathways [12]. However, the mechanism whereby PI3K activation by lithium mediates ventricular remodelling after MI is unknown. In contrast, previous studies have shown that lithium has an additive effect on cardiac hypertrophy in a model of abdominal aortic banding, a pathological hypertrophy [13]. The effect of lithium after MI on physiological compared with pathological hypertrophy is unknown. Lithium is highly toxic at regular doses and whether the subtherapeutic concentration is enough for optimal efficacy and acceptable toxicity remains controversial. Thus, the purpose of the present study was: (i) to investigate how lithium chloride (LiCl) at a low dose affects physiological or pathological hypertrophy during ventricular remodelling and (ii) to assess the axis of Akt/mTOR systems in a rat MI model.

## Materials and methods

All rats received humane care and the experiment was approved and conducted in accordance with local institutional guidelines of the China Medical University for the care and use of laboratory animals and conformed with the National Institutes of Health Guide for the Care and Use of Laboratory Animals*.*

### Animals

#### Part 1

Male Wistar rats (250–300 g) were intubated and the anterior descending artery was ligated using a 6-0 silk, resulting in infarction at the left ventricle (LV) as previously described [4]. For surgery, haemodynamics measurements, electrophysiological studies and sacrifice, rats were intraperitoneally anaesthetized with ketamine (90 mg/kg body weight (BW)) and xylazine (9 mg/kg). Anaesthesia monitoring was by rear-foot reflexes before and during procedures, observation of respiratory pattern and responsiveness to manipulations throughout the procedures. Twenty-four hours after ligation, rats were randomly assigned into either saline group (NaCl) or LiCl (1 mmol/kg per day). The drug was given orally by gastric gavage once a day. The drug was started 24 h after MI; during this window, the drug can maximize benefits while minimizing the possibility of a direct effect on infarct size [14]. For chronic lithium treatment, rats were given water and saline *ad libitum* to prevent hyponatraemia caused by lithium-induced increased excretion of sodium. To evaluate general toxicity of lithium, BW was monitored weekly. Mortality rate and general conditions of the animals were also observed daily throughout the whole experiment. The study duration was designed to be 4 weeks because the majority of the myocardial remodelling process in the rat (70–80%) is complete within 3 weeks [14]. Sham rats underwent the same procedure except the suture was passed under the coronary artery and then removed. Sham operation served as controls.

#### Part 2

Although results of the above study showed that LiCl significantly increased ventricular hypertrophy after infarction (see ‘Results’), the involved mechanism remained unclear. To rule out non-specific effect of lithium and confirm the importance of Akt and mTOR signalling in LiCl-induced hypertrophy, we employed deguelin (a specific Akt inhibitor) and rapamycin (an mTORC1 inhibitor) in an *ex vivo* experiment. Four weeks after induction of MI by coronary ligation, infarcted rat hearts were isolated and subjected to saline (NaCl), LiCl (0.4 mM) or a combination of LiCl and deguelin (10 μM, Sigma, St. Louis, MO) or LiCl and rapamycin (0.4 μM, Sigma, St. Louis, MO). Each heart was perfused with a non-circulating modified Tyrode’s solution as previously described [15]. Drugs were infused for 1 h. The doses of LiCl, deguelin and rapamycin used were as previously described [2,5,16]. At the end of the study, all hearts (*n*=5 per group) were used for Western blot of eukaryotic initiation factor 4E binding protein 1 (4E-BP1) and ERK in the remote zone (>2 mm outside the infarct).

#### Echocardiogram

At 28 days after operation, rats were lightly anaesthetized with intraperitoneal injection of ketamine (45 mg/kg) and xylazine (5 mg/kg). Echocardiographic measurements were done using the GE Healthcare Vivid 7 Ultra-sound System (Milwaukee, WI) equipped with a 14-MHz probe. M-mode tracing of the LV was obtained from the parasternal long-axis view to measure LV end-diastolic diameter dimension (LVEDD), LV end-systolic diameter dimension (LVESD) and fractional shortening (FS, %). The wall tension index (WTI) was defined as the ratio (LVEDD/2*posterior wall thickness) as described previously [17]. WTI was measured in order to indirectly assess myocardial wall stress. After this, the rats quickly underwent haemodynamic measurement after systemic heparinization.

#### Haemodynamics and infarct size measurements

Haemodynamic parameters and infarct size were measured in anaesthetized rats at the end of the study as described in detail in the Supplementary Material online.

#### Western blot analysis of Ser^473^-p-Akt1, Akt1, Thr^37/46^-p-4E-BP1, 4E-BP1, Thr^202^/Tyr^204^-p-ERK1/2 and ERK1/2

Samples were obtained from the remote zone at week 4 after infarction. Experiments were replicated three times and results were expressed as the mean value as described in detail in the Supplementary Material online.

The primary antibodies used were as follows: p-Akt1 (Ser^473^), p-4E-BP1 (Thr^37/46^), total-4E-BP1, p-ERK1/2 (Thr^202^/Tyr^204^) and total ERK1/2 antibody (Cell Signaling Technology, Beverly, MA) and Akt1 and β-actin (Santa Cruz Biotechnology, Santa Cruz, CA).

#### Real-time RT-PCR of GATA4, ANP, β-MHC and skeletal α-actin

mRNAs were quantified by real-time RT-PCR with cyclophilin as a loading control. The cardiac-specific transcription factor, *GATA4*, plays important roles in cardiac hypertrophy. For a detailed method, please refer to the Supplementary Material online.

#### Morphometric determination of myocyte size and interstitial fibrosis

Because ventricular remodelling after infarction is a combination of reactive fibrosis and myocyte hypertrophy, we measured cardiomyocyte sizes in addition to myocardial weight to avoid the confounding influence of non-myocytes on cardiac hypertrophy. For a detailed method, please refer to the Supplementary Material online.

#### Laboratory measurement

Blood samples were collected from rats at the end of the study from the ascending aorta and serum was separated by centrifugation for the estimation of lithium levels using an EEL-flame photometer.

The NFAT activity was analysed by ELISA according to the manufacturer’s instructions (TransAM NFAT Family Transcription Factor Assay Kit; Active Motif). Briefly, nuclear extracts were added to the wells of a 96-well plate that contained the immobilized oligonucleotide carrying an NFAT consensus site, 5′-AGGAAA-3′. Proteins bound to this immobilized oligonucleotide were detected by incubating with a primary antibody that recognizes active NFAT, followed by horseradish peroxidase–conjugated secondary antibody and were quantified by spectrophotometry at 450 nm with a reference wavelength of 650 nm.

Histological collagen results were confirmed by hydroxyproline assay adapted from Stegemann and Stalder [18]. The samples from remote areas were immediately placed in liquid nitrogen and stored at −80°C until measurement of the hydroxyproline content. The results were calculated as hydroxyproline content per weight of tissue.

#### Statistical analysis

Results were presented as mean ± S.D. Comparisons among groups were assessed for significance by one-way ANOVA. When significant differences were detected, individual mean values were compared by Bonferroni’s post hoc test (SPSS, version 18.0, Chicago, IL). Probability values were two-tailed and *P*<0.05 was considered to be statistically significant.

## Results

### Lithium affects ventricular remodelling

Differences in mortality rates between saline- and lithium-treated infarcted groups were not found throughout the study. Most of the mortalities occurred within the first hours after ligation, with deaths due to excessive infarction and arrhythmia. No animals died due to lithium treatment. Relative heart weights corrected for tibia length at the end of the experimental period (12 weeks of age) are presented in Table 1. Consistent with a previous study [19], the gain in BW in lithium-treated rats was less than that in the saline-treated rats despite there being no difference in weight at the start of the study. Four weeks after infarction, the infarcted area of the LV was very thin and was totally replaced by fully differentiated scar tissue. The weight of the LV inclusive of the septum remained essentially constant for 4 weeks between the two infarcted groups. The lung weight (LungW)/tibia ratio, an index of lung oedema, was significantly lower in the LiCl-treated infarcted group compared with that in the saline-treated infarcted group. The values of +dp/d*t* and –dp/d*t* were significantly higher in the LiCl-treated infarcted group compared with those in the saline-treated infarcted group. LV end-systolic pressure (LVESP), LV end-diastolic pressure (LVEDP) and infarct size did not differ between the two infarcted groups.

**Table 1:** Cardiac morphology, haemodynamics and serum lithium concentrations at the end of the study

	Sham		Infarction treated with	
Parameters	Saline	LiCl	Saline	LiCl
Number of rats	10	10	11	12
BW, g	418 ± 11	355 ± 17^*^	410 ± 13	328 ± 18^†^
Heart rate, bpm	393 ± 15	407 ± 14	410 ± 20	404 ± 16
LVESP, mm Hg	104 ± 5	105 ± 5	97 ± 8	96 ± 7
LVEDP, mm Hg	5 ± 2	5 ± 2	20 ± 6^*^	18 ± 6^*^
+dp/d*t*, mm Hg/s	7831 ± 285	7918 ± 312	2382 ± 265^*^	3182 ± 259^*†^
–dp/d*t*, mm Hg/s	6723 ± 302	6982 ± 267	2281 ± 287^*^	2871 ± 254^*†^
Infarct size, %	…	…	40 ± 3	41 ± 3
LVW/tibia, mg/cm	242 ± 20	245 ± 19	297 ± 21^*^	286 ± 22^*^
RVW/tibia, mg/cm	67 ± 12	62 ± 14	92 ± 14^*^	89 ± 15^*^
LungW/tibia, mg/cm	392 ± 31	381 ± 35	498 ± 32^*^	450 ± 29^*†^
Li, mM	…	0.35 ± 0.05	…	0.39 ± 0.06

Values are mean ± S.D. LVW, left ventricular weight; RVW, right ventricular weight. ^*^P<0.05 compared with respective sham; ^†^*P*<0.05 compared with saline-treated infarcted group.

To characterize the cardiac hypertrophy on a cellular level, morphometric analyses of LV sections were performed (Figure 1a). Compared with saline-treated sham, saline-treated infarcted rats showed structural changes such as increased cardiomyocyte sizes (Figure 1b-b'), consistent with LV remodelling. LiCl-treated infarcted rats had a further increase in cardiomyocyte size compared with saline-treated infarcted rats.

**Figure 1:** Western analysis of RhoA membrane fraction and cytosolic fraction from the border zone at day 3 after MI. **(a)** Representative Masson trichrome-stained section of a vehicle-treated heart at 4 weeks after infarction (blue colour, from 12 to 4 o’clock); Bar =2 mm. **(b)** Representative cardiomyocytes (magnification 400×) and quantitative analysis of the cardiomyocyte sizes in the remote zone. Staining with FITC-labelled wheat germ haemagglutinin of cross-sectional sections of myocardium; Bar =50 μm.** (c)** Representative sections from the remote area with Sirius Red staining (red, magnification 400×) at 4 weeks after infarction; Bar =50 μm. (S-Sa), saline-treated sham; (S-LiCl), LiCl-treated sham; (MI-Sa), saline-treated infarcted rat; (MI-LiCl), LiCl-treated infarcted rat. Each column and bar represents mean ± S.D. (*n*=5–6 per group). ^*^P<0.05 compared with saline-treated sham; ^†^*P*<0.05 compared with LiCl-treated sham; ^‡^*P*<0.05 compared with saline-treated infarcted group

Fibrosis of the LV from the remote area was examined in tissue sections after Sirius red staining, as shown in Figure 1c-c'. Compared with sham, infarcted rats treated with saline had significant increased fibrosis, as evidenced by increased collagen staining. The lithium-treated infarcted rats showed attenuated cardiac fibrosis compared with saline-treated infarcted rats. Measurement of hydroxyproline content mirrored the histological observation (3.26 ± 0.96% dry weight tissue in saline-treated infarcted rats compared with 2.48 ± 0.67% dry weight tissue in lithium-treated infarcted rats, *P*<0.05).

LV functional parameters were studied by echocardiography 28 days after surgical procedure (Table 2, Figure 2). Compared with sham-operated hearts, MI hearts showed structural changes such as increased LV diastolic and systolic diameters, consistent with LV remodelling. Both LVEDD and LVESD in rats with MI were significantly reduced by LiCl compared with saline (*P*<0.05). LV FS was significantly higher in the LiCl-treated infarcted group compared with saline. A significant decrease in WTI was observed in the LiCl-treated infarcted group compared with saline (*P*<0.05). These data were corroborated by the results that +dp/d*t* and –dp/d*t* were significantly improved in the LiCl-treated infarcted group compared with saline.

**Table 2:** Echocardiographic findings at the end of the study

	Sham		Infarction treated with	
Parameters	Saline	LiCl	Saline	LiCl
LVEDD, mm	5.6 ± 0.2	5.5 ± 0.2	8.9 ± 0.3^*^	8.5 ± 0.3^*†^
LVESD, mm	3.4 ± 0.1	3.5 ± 0.1	7.1 ± 0.2^*^	6.5 ± 0.2^*†^
LVPW, mm	1.4 ± 0.1	1.5 ± 0.2	1.9 ± 0.2^*^	2.1 ± 0.2^*^
FS, %	39 ± 2	36 ± 2	19 ± 3^*^	24 ± 3^*†^
WTI	2.01 ± 0.08	1.83 ± 0.07^‡^	2.34 ± 0.10^*^	2.02 ± 0.09^*†^

Values are mean ± S.D. Abbreviations are as in Table 1. LVPW, left ventricular posterior wall. ^*^P<0.05 compared with respective sham; ^†^*P*<0.05 compared with saline-treated infarcted group; ^‡^*P*<0.05 compared with saline-treated sham.

**Figure 2:** Representative M-mode image Representative M-mode image reveals a hypokinetic-to-akinetic anterior wall and LV dilation in the infarcted hearts treated with either saline **(c)** or LiCl **(d)**. There are markedly dilated LVEDD and LVESD in the saline-treated infarcted group compared with those in the LiCl-treated infarcted group.

### Lithium increases phosphorylation of Akt and 4E-BP1

Western blot showed that lithium treatment resulted in a significant increase (*P*<0.05) in relative p-Akt level of 32 ± 8% compared with 25 ± 4% for relative level of p-Akt in saline-treated infarcted rats (Figure 3). Treatment with LiCl enhanced the 4E-BP1 phosphorylation by 138% (*P*<0.01) in the infarcted rats compared with the saline-treated rats. This effect of lithium treatment on the levels of 4E-BP1 phosphorylation was completely blocked in the presence of deguelin or rapamycin (Figure 4), implying the axis of Akt/mTOR in regulating 4E-BP1 activity.

**Figure 3:** Western blot in an *in vivo* study (Part 1 experiment) Western blots show the expression of p-Akt, p-4E-BP1 and p-ERK. There was a significant increase in the levels of p-Akt and p-4E-BP1 in the LiCl-treated infarcted rats compared with the saline-treated infarcted rats. Bar graphs represent the quantitative analysis and difference in the expression of p-Akt and p-4E-BP1, after they were normalized with corresponding total proteins respectively, in arbitrary units. The values are mean ± S.D. (*n*=5–6 per group). Experiments were replicated three times and results expressed as the mean value. S, sham; Sa, saline. *P<0.05 compared with saline-treated sham; ^†^*P*<0.05 compared with LiCl-treated sham; ^‡^*P*<0.05 compared with saline-treated infarcted group.

**Figure 4:** Western blot in an *ex vivo* study (Part 2 experiment) Western blot analysis of 4E-BP1 and ERK to furthermore confirm the Akt and mTOR on kinase activity in homogenates of the LV from the remote zone in a rat-isolated infarcted heart model. A significantly increased p-4E-BP1 level is noted in the LiCl-treated group compared with that seen in the saline-treated group, which was attenuated after administering deguelin (a specific Akt inhibitor) and rapamycin (an mTORC1 inhibitor). The values are mean ± S.D. (*n*=5 per group). Experiments were replicated three times and results expressed as the mean value. *P<0.05 compared with saline-, LiCl-deguelin-, and LiCl-rapamycin-treated infarcted rats; ^†^*P*<0.05 compared with saline-treated infarcted rats.

### Lithium inhibits NFAT and ERK activities

As expected, MI significantly increased NFAT-dependent transcription compared with sham (Figure 5a). Lithium administration significantly reduced the NFAT activity by 21% (*P*<0.05) in the infarcted rats compared with the saline-treated rats. These data indicate that a low concentration of lithium is efficient at selectively inhibiting important regulators involved in pathological hypertrophy (such as NFAT).

**Figure 5:** NFAT activity and RT-PCR of *GATA4*, *ANP, β-MHC* and *skeletal α-actin* Each mRNA was corrected for an mRNA level of cyclophilin. Each column and bar represents mean ± S.D. ^*^P<0.05 compared with saline-treated sham; ^†^*P*<0.05 compared with LiCl-treated sham; ^‡^*P*<0.05 compared with saline-treated infarcted group.

In addition, the MI-induced up-regulation of the p-ERK levels was attenuated in the presence of lithium (Figure 3).

Finally, to further assess the role of Akt/mTOR pathway in lithium-attenuated p-ERK levels, Western blot was performed on infarcted hearts treated with deguelin or rapamycin in an *ex vivo* model. As shown in Figure 4, neither deguelin nor rapamycin affected the ERK phosphorylation compared with lithium alone, implying the attenuated ERK levels after adding lithium is not related to Akt/mTOR pathway.

### Lithium inhibits GATA4 expression and foetal gene expressions of ANP, β-MHC and skeletal α-actin

MI increased gene expressions of *GATA4, ANP, β-MHC* and *skeletal α-actin* (Figure 5b–e), as expected. Saline-treated infarcted hearts were found to significantly increase *GATA4* expression as compared with saline-treated sham (1.28 ± 0.11 compared with 0.76 ± 0.15 in sham, *P*<0.05, Figure 3). LiCl treatment in post-infarcted hearts resulted in a decrease in *GATA4* compared with saline treatment. The foetal gene expressions of *ANP, β-MHC* and *skeletal α-actin* showed similar changes to *GATA4*.

## Discussions

Our data indicate for the first time that lithium at a low dose could be utilized to alleviate the pathological development of hypertrophy and improve adaptive physiological cardiac growth. These results were concordant for beneficial effects of lithium, as documented structurally by increase in myocyte sizes, molecularly by myocardial Akt/4E-BP1 levels and functionally by improvement of cardiac contractility. Our results were consistent with previous observation that enhanced PI3K activity by pharmacological intervention that had a beneficial impact against subsequent pressure overload by inhibiting pathological processes [20]. Thus, lithium acts as an activator of physiological hypertrophy and inhibited pathological hypertrophy.

The present study provides several novel findings that increase our understanding of the signal transduction mechanism of the cardioprotection afforded by ventricular remodelling. A low dose of lithium is efficient at selectively inhibiting regulators involved in pathological hypertrophy (such as NFAT, ERK and GATA4), while enhancing pathways involved in physiological hypertrophy (Akt and 4E-BP1) as evidenced by three observations (Figure 6).

### Lithium shows beneficial effects at a low dose

Recommendations for target serum lithium concentrations (0.8–1.2 mM) appear to have been originally derived from studies of the effect of lithium on various indexes such as mania recurrence [21]. Despite the obvious advantages of chronic lithium therapy, its clinical use is often curtailed by its narrow therapeutic index and its devastating overdose-induced toxicity. Furthermore, it should be noted that in spite of therapeutic lithium serum levels, wide variations between serum lithium levels and intracellular concentrations of lithium have been reported [22,23]. However, low dose levels have scantly been assessed in animal and clinical studies. The present study showed lithium at a low dose can provide beneficial biological effects after MI.

### Lithium enhances physiological remodelling

Both lithium- and infarction-induced hypertrophy are associated with an increase in myocyte size but with distinct molecular and histological phenotypes. During ventricular remodelling after MI, pathological cardiac hypertrophy is characterized molecularly, by the induction of foetal genes, such as *ANP*, *β-MHC* and *skeletal α-actin*; histologically, by increased interstitial fibrosis and left ventricular dilatation; and functionally, by impaired cardiac contractility. Given the reduction in LV dilatation, better-preserved systolic function, reduction in WTI and decreased expression of foetal genes in the lithium treatment, this hypertrophy may be viewed as more ‘physiological’ than ‘pathological’.

**Figure 6:** Signalling cascades leading to physiological and pathological hypertrophy after infarction The diagram summarizes the histological, molecular and pharmacological evidence. Inhibition of these signalling pathways by their respective inhibitors is indicated by the vertical lines. Our data suggest that lithium is efficient at selectively inhibiting important regulators involved in pathological hypertrophy (such as NFAT and ERK), while augmenting pathways involved in physiological hypertrophy (such as 4E-BP1).

Given p-4E-BP1 is activated in the development of physiological hypertrophy, lithium-increased p-4E-BP1 levels are blunted to the level similar to the vehicle group when Akt1 is inhibited by deguelin, implying that Akt is essential for the development of physiological hypertrophy. Previously, Chun et al. [24] reported that deguelin treatment had only mimimal effects on the MAPK pathway. In our study, we also found no significant differences in phosphorylation levels of ERK, suggesting that deguelin application does not have a sufficient effect on MAPK signalling after MI.

Whether Akt-induced cardiac hypertrophy is physiological or pathological is complex [17]. Activation of PI3K/Akt1 signalling is required for exercise-induced hypertrophy [16]. Others also point out that Akt1 is a critical mediator of pathological cardiac hypertrophy [25,26]. These latter conclusions, however, are derived from transgenic mouse models overexpressing constitutively active Akt1 at 15-fold higher than the physiological levels. Overexpression of Akt1 to this extent can overtake the function of other Akt isoforms and also can lead to off-target effects because of non-physiological protein–protein interactions and aberrant intracellular localization. Indeed, Akt1 has a dichotomous role in cardiac remodelling by mediating physiological compared with pathological signalling based upon the duration, the intensity and the type of stress. Our study answered the question of the effect of chronic pharmacological activation of Akt with lithium on cardiac hypertrophy after MI.

Our results do not seem consistent with previous studies, showing that chronic Akt1 activation, which activates mTORC1, has been shown to worsen aging-induced cardiac hypertrophy and impair myocardial contractile [27]. mTOR exerts its main cellular functions by interacting with specific adaptor proteins to form two distinct multiprotein complexes, mTORC1 and mTORC2 [28]. mTORC1 has been shown to play a crucial role in the regulation of cellular homoeostasis, growth and response to stress. However, its functional role is still under debate because different roles of mTORC1 have been suggested under various experimental conditions. The data from the pharmacological modulators of mTOR and the animal models with genetic modifications of the components of mTOR signalling pathway will be expected to be different because the degree of mTORC1 activation among models is different. The degree of mTORC1 activation and the mTORC1 physiological functions to be preserved to convert mTORC1 activation from detrimental into beneficial during cardiac stress remains unclear. Indeed, our results were consistent with the previous findings, showing that the activation of mTORC1/4E-BPs axis plays a role in physiological hypertrophy [29].

### Lithium inhibits pathological remodelling

PI3K pathway can inhibit pathological growth in addition to promoting physiological growth. Akt is activated by PI3K (p110α) to induce physiological hypertrophy but is also activated in response to GPCR agonists, e.g. endothelin-1 via another PI3K isoform (p110γ) that induces pathological hypertrophy [2]. That is why the p-Akt levels were significantly higher after inducing MI (Figure 3). Furthermore, PI3K (p110α) signalling negatively regulated GPCR-stimulated extracellular responsive kinase and Akt (via PI3K, p110) activation [16]. Thus, although there was similar activation of Akt between the two groups of lithium-treated sham rats and vehicle-treated infarcted rats, we assessed ERK1/2 activation. p-ERK was significantly increased in infarcted hearts but not changed in the lithium-treated sham, implying different downstream signalling pathways. Finally, in the infarcted rats, lithium administration reduced the p-ERK levels and NFAT activity compared with the saline group, implying the inhibitory effect of lithium on pathological hypertrophy. Our results were consistent with the notion that the PI3K/Akt axis is more linked to physiological hypertrophy, whereas MAPK signalling, in collaboration with the NFAT pathway, participates in the development of the pathological hypertrophy [30].

To more directly address this interpretation, molecular markers of pathological cardiac hypertrophy were analysed by mRNA. The data showed that ventricular remodelling was associated with the expression of *ANP*, *β-MHC* and *skeletal α-actin* in the heart. Dephosphorylated NFAT (increased activity) enters the nucleus where it interacts with GATA4 and causes transcriptional activation of hypertrophic foetal genes leading to cardiomyocyte hypertrophy [31]. These foetal gene expressions are inhibited after lithium administration, consistent with the results that lithium inhibited pathological remodelling.

### Other mechanisms

Although the present study suggests that the mechanisms of lithium-induced physiological ventricular remodelling may be related to an Akt/mTOR axis, other pathways may take part in the effect of lithium. It may be supposed that lithium elicits cardioprotection, in part, through its ability to inhibit GSK-3β by increasing GSK-3β phosphorylation. Previous studies have shown that the lack of GSK-3β phosphorylation in response to pressure overload is associated with reduced hypertrophy and development of dilated cardiomyopathy, highlighting the important role of GSK-3β phosphorylation in the development of compensatory hypertrophy [32]. Thus, lithium may increase physiological cardiac hypertrophy by inhibiting GSK-3β activity.

### Clinical implications

The present study was undertaken to explore the possibility that lithium might have clinical efficacy for the treatment after MI. Traditional therapeutics to prevent post-MI remodelling (e.g. angiotensin-converting enzyme inhibitors and angiotensin-receptor antagonists) are effective to some degree but progression to congestive heart failure or death, despite standard approaches, is common. Novel signalling pathways involved in the cardiac remodelling after MI, like Akt/mTOR signalling, need to be explored. Induction of physiological cardiac hypertrophy may be a potential therapeutic strategy for the treatment of heart failure. Lithium’s ability to induce hypertrophy would reduce LV WTI according to Laplace’s law, and its effects on contractility would enhance the function of the non-infarcted myocardium, both of which would be of particular benefit if applied, while the process of remodelling was beginning. Our findings may have potential implications as a therapeutic agent for treatment of patients post-MI. Activation of PI3K (p110α), via exercise training or pharmacological approaches, offers a novel therapeutic strategy for preventing LV remodelling in patients at the risk of developing heart failure. While angiotensin converting enzyme inhibitors and angiotensin receptor blockers slow LV remodelling by targeting pathological hypertrophy signalling pathways, activation of PI3K (p110α) attenuates LV remodelling by activating physiological hypertrophy signalling pathways as well as inhibiting pathological signalling pathways.

### Study limitations

There are some limitations in the present study that have to be acknowledged. First, our studies on PI3K/Akt signalling were obtained by pharmacological inhibition. Thus, we can not exclude the non-specific actions of drugs. Second, lithium may affect the serum sodium levels [33] and subsequently modulate the hypertrophy. We did not measure the serum sodium levels. The LiCl administration regulates serum sodium levels in a dose-dependent manner [33]. Previous studies have shown in rats that chronic administration of LiCl at the dose of 50  mg/kg per day, higher than that used in the present study (1 mmol/kg per day of LiCl, equivalent to 42 mg/kg per day), did not significantly change the serum sodium levels [33]. Thus, although we did not measure the sodium levels, it is logical to speculate that the serum sodium levels would not significantly change at the subtherapeutic dose.

In conclusion, our findings suggest that in the setting of MI, a dysbalance towards pathological pathways occurs and leads to a deterioration of cardiac remodelling and function, which can be corrected by lithium administration through an Akt/mTOR pathway. Lithium may constitute a new therapeutic option for mending the infarcted myocardium and its clinical efficacy needs to be tested in clinical trials.

## Abbreviations

ANP: atrial natriuretic peptide
BW: body weight
ERK: extracellular-signal-regulated kinase
ERK1/2: extracellular-signal-regulated kinase 1/2
FS: fractional shortening
GPCR: G-protein-coupled receptor
LiCl: lithium chloride
LungW: lung weight
LV: left ventricle
LVEDD: LV end-diastolic diameter dimension
LVEDP: LV end-diastolic pressure
LVESD: LV end-systolic diameter dimension
LVESP: LV end-systolic pressure
MAPK: mitogen-activated protein kinase
MI: myocardial infarction
mTOR: mammalian target of rapamycin
NFAT: nuclear factor of activated T-cells
PI3K: phosphoinositide 3-kinase
WTI: wall tension index
4E-BP1: eukaryotic initiation factor 4E binding protein 1
β-MHC: β-myosin heavy chain
